RETRACTED

# DNA-PK_CS_ binding to p53 on the *p21^WAF1/CIP1^* promoter blocks transcription resulting in cell death

**DOI:** 10.18632/oncotarget.378

**Published:** 2011-12-20

**Authors:** Richard Hill, Patricia A. Madureira, David. M. Waisman, Patrick W.K. Lee

**Affiliations:** ^1^ Department of Microbiology & Immunology, Dalhousie University, Halifax, Nova Scotia, Canada; ^2^ Department of Biochemistry and Molecular Biology, Dalhousie University, Halifax, Nova Scotia, Canada; ^3^ Department of Pathology, Dalhousie University, Halifax, Nova Scotia, Canada

**Keywords:** DNA-PKCs, p53, p21 transcription suppression

## Abstract

A key determinant of p53-mediated cell fate following various DNA damage modalities is *p21^WAF1/CIP1^* expression, with elevated *p21* expression triggering cell cycle arrest and repressed *p21* expression promoting apoptosis. We show that under pro-death DNA damage conditions, the DNA-dependent protein kinase (DNA-PK_CS_) is recruited to the *p21* promoter where it forms a protein complex with p53. The DNA-PK_CS_-associated p53 displays post-translational modifications that are distinct from those under pro-arrest conditions, ablating *p21* transcription and inducing cell death. Inhibition of DNA-PK activity prevents DNA-PK_CS_ binding to p53 on the *p21* promoter, restores *p21* transcription and significantly reduces cell death. These data demonstrate that DNA-PK_CS_ negatively regulates p21 expression by directly interacting with the *p21* transcription machinery via p53, driving the cell towards apoptosis.

## INTRODUCTION

The most prevalent reported genetic defect observed in human cancer is the loss or inactivation of the tumor suppressor protein p53 [1, 2]. In unstressed cells, p53 is maintained at a low level by its negative regulator MDM2 [3, 4] and is at the center of a complex signalling network. In response to a broad range of oncogenic stresses including DNA damage, chemical exposure or hypoxia, p53 can facilitate either DNA repair (promoting cell survival) or trigger apoptosis (programmed cell death), thereby ensuring the removal of irreparably damaged cells. p53 is able to dictate these cell fates in large measure because it is a transcription factor with sequence-specific DNA-binding activity that regulates the expression of a plethora of genes [5]. Chromatin-immunoprecipitation (ChIP) studies revealed that p53 directly binds to approximately 1600 genes that fall primarily into three categories: cell cycle inhibition, apoptosis, and genome stability [6]. Despite this wealth of information, the mechanism regarding how p53 mediates the choice between life and death remains unclear.

The generally accepted dogma for p53-controlled cell fate holds that cell cycle arrest is predominantly mediated by the expression and activation of the cyclin-dependent kinase inhibitor CDKN1A (p21) [7-9], in contrast to apoptosis that is primarily controlled by the expression and activation of pro-apoptotic genes including *Bax* [10] and *PUMA* (p53 upregulated modulator of apoptosis) [11, 12]. While p21's ability to inhibit both the G_1_-S and the G_2_-M cell cycle transitions is well established, emerging evidence suggests that p21 also possesses potent anti-apoptotic activity to complement its pro-arrest functions. For example, it has been shown that p21 binds to and inactivates procaspase 3, thereby inhibiting apoptosis [13]. In addition, caspase 2, which acts upstream of caspase 3, is transcriptionally repressed by p21 [14]. Furthermore, p21 can also suppress the induction of pro-apoptotic genes by MYC or E2F1 by direct inhibition of their transcription functions [15]. There is also evidence that p21 protects cells from irradiation-induced apoptosis by blocking CDKs involved in the activation of the caspase cascade downstream [16] while nutrient starvation induced cell death is also suppressed by p21 [17]. Collectively, these data suggest that p21 is capable of launching a multi-level anti-apoptosis strategy, effectively counteracting the pro-apoptotic functions of Bax and PUMA. Thus, while the induction and presence of pro-apoptotic genes are required for the cell to trigger a potent apoptotic response, there is also the absolute requirement for the cell to abolish p21 expression and mediate p21 protein degradation to enable apoptosis to proceed.

RETRACTED

Since both pro-arrest (*p21*) and pro-death (e.g. *Bax* and *PUMA*) elements are downstream transcriptional targets of p53, the delicate balance between their expression levels necessarily hinges on the selective activation or suppression of specific p53 transcriptional activity [18-22]. In this regard, post-translational modifications of p53 have been shown to play a central role. Depending on the nature of DNA damage or cell stress, p53 undergoes different modifications that dictate its ultimate function. A most common and critical modification of p53 is ser15 phosphorylation that prevents MDM2-mediated monoubiquitination and nuclear export, allowing p53 to accumulate in the nucleus [4]. The ser46 and ser315 residues have also attracted significant attention as following ser46 phosphorylation, p53 specifically induces pro-apoptotic gene expression [23, 24] in contrast to ser315 phosphorylation that stimulates the expression of *p21* [25]. In addition to phosphorylation, acetylation of p53 has also been shown to regulate p53-dependent transcription (for a review see [26]. The acetylation of lys120 was shown as an absolute requirement for *PUMA* and *Bax* transcription after p53 promoter recruitment. In contrast, lysine 382 acetylation specifically and significantly increased *p21* expression [27, 28]. Based on these studies, it is clear that there is enormous complexity regarding p53 posttranslational modifications, that many appear to be stress-specific, and that these diverse modifications can activate or repress select target genes dictating cell fate.

RETRACTED

The phosphatidylinositol 3-kinase-like protein kinases (PI3KKs) are large proteins that include Ataxia telangiectasia mutated (ATM), ATM and Rad3-related (ATR), and the DNA-dependent protein kinase (DNA-PK) that are each activated following a range of cellular stresses and can direct p53 posttranslational modifications. The most defined cellular response is the activation of the G_1_ and G_2_ cell cycle checkpoints mediated by ATM via p53 phosphorylation that leads to *p21* transcription and cell cycle arrest [29, 30]. ATR reinforces this response by the phosphorylation of signaling intermediates including checkpoint kinase 1 (Chk 1) [31]. The most classically defined DNA-PK function is V(D)J recombination that is responsible for antibody diversity and normal immune development (reviewed in [32, 33]). In addition to this well characterized role, however, there is now a significant body of data implicating DNA-PK_CS_ as an upstream element of p53, being involved in the latter's posttranslational modification and apoptotic response to severe DNA damage [20, 34-37]. It thus appears that ATM/ATR and DNA-PK play antagonistic roles in dictating stress-induced cell fate (cell cycle arrest *vs* apoptosis) through their control of a common element, p53 [38, 39]. More recent data suggest that it is the control over p53-mediated *p21* expression that ultimately determines cell fate, with ATM/ATR and DNA-PK promoting and suppressing *p21* expression, resulting in cell cycle arrest and apoptosis, respectively [40-43].

With DNA-PK's emerging role as an important mediator of apoptosis, it is important to understand how DNA-PK activation could lead to down-regulation of p21. Here we report that under conditions that favor cell death, DNA-PK_CS_ forms a protein complex with p53 and is recruited to the *p21* promoter. This complex formation abrogates *p21* transcription, preventing cell cycle arrest and as a result sets into motion a potent apoptotic response to DNA damage. DNA-PK_CS_ does not inhibit the ability of p53 to bind to target gene promoters (pro-arrest or pro-death), however, only the transcription of the pro-arrest *p21* gene is blocked. DNA-PK_CS_ therefore directly interferes with the p53-mediated *p21* transcription machinery, priming the cell for apoptosis.

RETRACTED

## RESULTS

### p21 expression correlates with cell fate following DNA damage

To investigate how p53 can direct cell fate we exposed cells to various DNA damaging conditions that result in cell cycle arrest, apoptosis, or both. Gemcitabine is a chemotherapeutic and an analog of deoxycytidine that inhibits DNA synthesis [44]. Doxorubicin is a chemotherapeutic anthracycline that creates DNA breaks via the inhibition of topoisomerase II [45]. Chromium (VI) is a carcinogen that binds DNA, generating adducts, single and double strand DNA breaks [46], while γ−irradiation (IR) introduces double strand DNA breaks. All four of these DNA damaging agents activated and induced significant accumulation of the p53 protein (Fig. 1A and S1A), however, their effects on cell fate were very different. Whereas chromium treatment triggered significant apoptosis but no cell cycle arrest (measured by caspase-3 cleavage and the accumulation of a sub-G_1_ cell population), IR induced almost exclusively cell cycle arrest (with little to no apoptosis) (Fig. 1A, 1B and S1B). The effects of gemcitabine and doxorubicin fell between the two ends of the spectrum, with gemcitabine inducing significantly less cell cycle arrest than doxorubicin. These four agents therefore provided a full cell fate spectrum that allowed us to more precisely characterize the role of DNA-PK_CS_ in directing p53-dependent cell fate.

**Figure 1:** All DNA damage modalities induce p53 but manifest different p21 expression levels that correlate with cell cycle arrest or apoptosis (A) [*p53*^+/+^] HCT116 cells were exposed to chromium (Cr(VI)), gemcitabine (Gem), doxorubicin (Doxo) or γ-irradiation (γ-IR) for the specified times (hr). Cell extracts were subjected to immunoblot analysis for p53, caspase-3 or β-actin expression. (B) HCT116 *p53*^+/+^ cells were exposed to Cr(VI), Gem, Doxo or γ-IR. At the time points indicated DNA content was analyzed by flow cytometry of cells stained with BrdU and propidium iodide. Each plot represents the cell cycle profile at 24 h post damage. Quantification of the percentage of the sub-G_1_, G_1_ and G_2_ DNA content was determined for each sample and is represented in each graph (20,000 total events counted). (C) HCT116 *p53*^+/+^ cell extracts were subjected to immunoblot analysis for p21, MDM2, PUMA, Bax, and β-actin expression. (D) Trizol RNA extraction was carried out from [*p53*^+/+^] HCT116 cells 12 h post damage; cDNA was generated and the expression level for *p21* was measured. The mRNA expression levels were normalized to *GAPDH* mRNA, and are represented as fold increase or decrease over untreated cells. Error bars represent the standard deviation obtained from three independent experiments.

RETRACTED

We then investigated the protein expression of key p53-regulated genes over time following exposure to each agent in a range of classically studied model cancer cell lines. As exemplified by the [*p53*^+/+^] HCT116 cell line, the most dramatic difference between the four treatments was noted for p21 expression (Fig. 1C). Whereas IR and doxorubicin treatments resulted in the gradual accumulation of p21, chromium and gemcitabine caused a significant reduction of the protein at 6 and 12 h post damage. In contrast to p21, the total protein levels of MDM2, PUMA and Bax were equivalently induced by each modality investigated. The reduced p21 protein levels post gemcitabine or chromium treatment corresponded with the lowered transcription of this gene (Fig. 1D and S1C) as these agents had no effect on protein stability or the half-life of the p21 transcript [20]. Collectively, our results are compatible with the view that the reduction in p21 expression allows continued cell cycle progression which, in the presence of both DNA damage and the continuous expression of apoptotic proteins, ultimately leads to cell death.

### Post-translational modifications of p53 bound to the p21 promoter

We next questioned whether p53 was recruited to the promoters of *p21* under each DNA damage modality even where expression of this gene was suppressed. Accordingly, chromatin immunoprecipitation (ChIP) assays were carried out and revealed surprisingly that p53 was recruited to both the distal and proximal *p21* promoters irrespective of whether there was active *p21* gene transcription (Fig. 2 (top panel) and S1D). To determine if the p53 bound to the *p21* promoters was modified differently following each DNA damage regime, ChIP analyses were performed using a panel of antibodies against specific modified p53 residues. The results (Fig. 2 and S2) show that while all *p21* promoter-bound p53 was phosphorylated on ser15 following exposure to any of the four DNA damage agents, enhanced ser37 phosphorylation was found primarily on p53 bound to the *p21* promoters under conditions (chromium or gemcitabine) that instigated cell death. Conversely, phospho-ser315 and acetyl-lys382 were found mainly on *p21* promoter-bound p53 under pro-arrest (doxorubicin or IR) conditions. These results clearly indicate that depending on the DNA damage modality, the p53 bound to the p21 promoters was modified differently, leading to either active *p21* transcription (mediating cell cycle arrest), or *p21* transcription repression (resulting in cell death).

RETRACTED

**Figure 2:** *p21* promoter-bound p53 is differently modified under arrest versus apoptotic conditions Chromatin immunoprecipitation (ChIP) was carried out with [*p53*^+/+^] HCT116 cells following mock or 6 h post DNA damage with the indicated modalities using the total or isoform-specific anti-p53 antibodies indicated. PCR was performed for either the distal (-2.2 kb) *p21* or proximal (-1.3 kb) *p21* promoter regions. Quantification of the bands following each DNA damage modality was determined in triplicate and represented for each promoter region. Error bars in all panels represent the standard deviation obtained from three independent experiments.

While we primarily focused on the *p21* promoters, we also examined p53 modifications on the *MDM2*, *PUMA* and *Bax* promoters under each DNA damage condition (Fig. S3). Our results show that p53 phosphorylated at ser15 was found on the *MDM2* promoter at 6 h post damage under all DNA damage conditions, but was bound to the *PUMA* promoter only under conditions that induced cell death (chromium or gemcitabine) and only bound to the *Bax* promoter following Cr(VI) exposure. Interestingly, p53-ser37 could be detected on both the *MDM2* and *PUMA* promoters 6 h post chromium, gemcitabine or doxorubicin exposure. No p53-ser37 could be detected on the *Bax* promoter following exposure to any of our DNA damage agents. In contrast to other p53 modifications, we noted the enhanced recruitment of p53-phopho-ser33 and phosphor-ser46 isoforms to all the promoters examined 6 h post damage with any of our tested agents. Collectively, these results indicate that for each p53-dependent cell phenotype (pro-arrest or cell death) there are significantly different p53 post translational profiles.

### Autophosphorylated DNA-PK_CS_ and p53 form a protein complex under pro-apoptotic conditions

Having noted distinct p53 post-translational modifications (phosphorylation/acetylation) following DNA damage that triggered cell cycle arrest or cell death (due to continued cycling of DNA damaged cells) correlated with disparate *p21* promoter recruitment and expression, we questioned which upstream activators of p53 mediated this response. We examined the three major PI3KK's ATM, ATR and DNA-PK_CS_ since they dictate specific p53 responses linked primarily to either the induction of cell cycle arrest (ATM/ATR) or apoptosis (DNA-PK_CS_). We found that all three PI3KKs are activated (phosphoryation at ser1981 for ATM, ser428 for ATR, and thr2609 for DNA-PK_CS_) under any of the four DNA damage conditions (Fig. 3A and S4A). As expected, all ATM and ATR phosphorylations were inhibited by the ATM/ATR-specific inhibitor, CGK-733 [47], but not by the DNA-PK-specific inhibitor, NU-7026 [48]. However, the use of these inhibitors on DNA-PK_CS_ thr2609 phosphorylation was revealing. It clearly showed that depending on the DNA damage treatment used, this phosphorylation event was dictated by different PI3KKs. The DNA-PK inhibitor NU-7026 effectively blocked thr2609 phosphorylation under pro-death (chromium and gemcitabine) conditions, but not under pro-cell cycle arrest (doxorubicin and IR) conditions. Conversely, the ATM/ATR inhibitor CGK-733 did not block thr2609 phosphorylation under damage conditions that lead to cell death (chromium or gemcitabine) but its inhibitory effect, albeit partial, under pro-arrest conditions (doxorubicin or IR) was evident. Our results show that the DNA-PK_CS_ phosphorylated (likely via autophosphorylation) under DNA damage conditions that lead to cell death is intrinsically different from the DNA-PK_CS_ activated (via ATM/ATR [49]) under cell cycle arrest conditions. This raises the hypothesis that DNA-PK_CS_ activated under certain damage conditions is destined to induce cell death by the suppression of cell cycle arrest, whereas DNA-PK_CS_ activated under pro-arrest conditions is poised to perform its DNA repair duty following cell cycle arrest.

RETRACTED

**Figure 3:** DNA-PK_CS_ activation under pro-apoptotic conditions is independent of ATM/ATR and forms a complex with p53 (A) [*p53*^+/+^] HCT116 cells were pre-incubated with the DNA-PK inhibitor NU-7026 (10 μM) or the ATM/ATR inhibitor CGK-733 (20 μM) and exposed to Cr(VI), Gem, Doxo or γ-IR for 12 h. Cell extracts were prepared and subjected to immunoblot analysis for total DNA-PK_CS_ or P-thr2609 DNA-PK_CS_. (B) The cell extracts from (A) were subjected to immunoblot analysis for total p53. (C) [*p53*^+/+^] HCT116 cells were exposed to Cr(VI), Gem, Doxo or γ-IR for the specified times. Cell extracts were prepared, immunoprecipitated (IP) with an anti-DNA-PK_CS_ or anti-p53 antibody, and subjected to western blot (WB) analysis for p53 or DNA-PK_CS_. Immunoblots for total p53 and total DNA-PK_CS_ in the extracts are also shown. (D) (*left*) Extracts prepared from 12 h post damage cells were immunoprecipitated with an anti-DNA-PK_CS_ antibody and analyzed for co-precipitated specific p53 isoforms. (*Right*) Extracts from [*p53*^−/−^] HCT116 cells were used to confirm antibody specificity.

The specific activation of ATM/ATR and DNA-PK under pro-death and pro-arrest conditions following each DNA damage regime was also reflected by their specific action on p53. Fig. 3B and S4B show that the ATM/ATR inhibitor effectively blocked p53 accumulation under pro-arrest conditions, but not under conditions that actuated cell death. Conversely, the DNA-PK inhibitor blocked p53 accumulation under pro-death DNA damage conditions (in the absence of cell cycle arrest) but not under pro-arrest conditions. Thus, p53 accumulation under pro-death or pro-arrest conditions is dependent on DNA-PK_CS_ or ATM/ATR, respectively. This is again consistent with the observation that p53 is modified differently under the two cell phenotypes.

RETRACTED

To further support this observation, we have previously shown that murine cell lines expressing adenovirus E1A (thus are unable to induce cell cycle arrest) undergo cell death post irradiation and that DNA-PK_CS_ and p53 form a protein-protein complex [34]. To determine if this complex formation occurs in human lines and correlates strictly with cell death, co-immunoprecipitation was carried out on lysates from cells damaged under the four DNA damage conditions. We found that both gemcitabine and chromium induced the formation of a DNA-PK_CS_/p53 protein complex that was not detected following doxorubicin treatment or IR (Fig. 3C and S4C). These observations, together with the results shown in Fig. 3B, raise the hypothesis that p53/DNA-PK_CS_ only form a protein/protein complex following DNA-PK_CS_ autophosphorylation and that when DNA-PK_CS_ is phosphorylated by ATM/ATR this protein complex does not form. In addition, the p53 bound to DNA-PK_CS_ was found to be phosphorylated on ser15, ser37, and ser46, and acetylated at lys120, in agreement with our ChIP studies (Fig. 3D). It is noteworthy that all of these modifications have been strongly linked with enhancing p53-dependent apoptosis [24]. Furthermore and consistent with our ChIP data, we were unable to detect phospho-ser315 or acetyl-lys382 p53 in the DNA-PK/p53 complex.

### DNA-PK_CS_/p53 interaction occurs on the p21 promoter

The observation that *p21* promoter-bound p53 and p53 bound in a complex with DNA-PK_CS_ are similarly modified led us to hypothesize that DNA-PK_CS_ could be recruited to the *p21* promoters under pro-death DNA damage conditions. This was indeed found to be the case. We noted the rapid binding of DNA-PK_CS_ to both distal and proximal *p21* promoters under pro-death (DNA damage conditions chromium or gemcitabine) but not pro-arrest conditions (doxorubicin or IR) in a range of model cancer cell lines (Fig. 4A, S5A and S5B). This recruitment was p53-dependent as we could not detect significant DNA-PK_CS_ binding to the *p21* promoters in similarly treated *p53*^−/−^ HCT116 cells, and no DNA-PK_CS_ binding was observed on the GAPDH promoter that was used throughout as our negative control. It is noteworthy that DNA-PK_CS_ recruitment to the *PUMA* and *Bax* promoters was negligible relative to the *p21* promoters (Fig. 4A), and could only be detected at late time points (24 h after chromium exposure or 48 h post gemcitabine treatment) once the cellular phenotype was markedly apoptotic. As expected, the *p21* promoters-bound DNA-PK_CS_ was found to be phosphorylated at thr2609 (Fig. 4B, S5A and S5B).

RETRACTED

**Figure 4:** DNA-PK_CS_ forms a complex with p53 on the p21 promoters under pro-apoptotic conditions (A) ChIP was carried out with [*p53*^+/+^] HCT116 cells following mock or 6 h post DNA damage with the indicated modalities using the anti-DNA-PK_CS_ antibody. PCR was performed for both the distal (-2.2 kb) *p21* and proximal (-1.3 kb) *p21* promoter regions. Quantification of the bands following each DNA damage modality was determined for triplicate studies and represented for each promoter region. (B) ChIP assays were conducted as in (A) using an anti-P-thr2609-DNA-PK_CS_ antibody. (C) Top left: ChIP assay for p53 from [*p53*^+/+^] HCT116 cells 6 h post Cr(VI), Gem, or γ-IR exposure. Top right: ChIP assay for p53 from [*p53*^+/+^] HCT116 cells following DNA-PK_CS_ immunodepletion. Bottom left: ChIP assay for DNA-PK_CS_ 6 h post DNA damage. Bottom right: ChIP assay for DNA-PK_CS_ following p53 immunodepletion. PCR was performed for the distal (-2.2 kb) and the proximal (-1.3 kb) *p21* promoter regions. The error bars in all panels represent standard deviation obtained from three independent experiments.

To demonstrate that DNA-PK_CS_ recruited to the *p21* promoters represented the same population that was associated with p53, we carried out immune-depletion experiments followed by ChIP analysis. Under conditions where *p21* transcription was repressed following chromium or gemcitabine treatment, immune-depletion of nuclear lysates with an anti-DNA-PK_CS_ antibody led to the drastic reduction of p53 bound to the *p21* promoters (Fig. 4C). This was not observed with nuclear lysates from IR-treated cells. Conversely, reciprocal immune-depletion with an anti-p53 antibody effectively removed DNA-PK_CS_ bound to the *p21* promoters following chromium or gemcitabine treatment while no DNA-PK_CS_ could be detected on these promoters following IR treatment. Taken together, these studies clearly demonstrate that p53 and DNA-PK_CS_ form a protein complex and that this complex is localized to the *p21* promoter.

We next compared the temporal kinetics of p53 and DNA-PK_CS_ recruitment to the *p21* promoters. As revealed by ChIP analysis, the recruitment of p53 on the proximal and distal *p21* promoter was detected as early as 30 min post DNA damage (gemcitabine or chromium) on the distal *p21* promoter and 3 h on the proximal promoter (Fig. 5A, 5B, 5D and 5E). A similar recruitment profile was also observed in the Panc-1 cell line (Fig. S6A, S6B, S6C and S6D). In contrast, the temporal recruitment of DNA-PK_CS_ was significantly slower than p53, with DNA-PK_CS_ binding first detected on the distal *p21* promoter around 3 h and on the proximal promoter approximately 6 h post damage. This shows that p53 recruitment to both *p21* promoters precedes that of DNA-PK_CS_, suggesting that the early recruitment of p53 to the *p21* promoters is likely independent of DNA-PK.

RETRACTED

**Figure 5:** p53 recruitment to the p21 promoter precedes DNA-PK_CS_ binding (A) ChIP assay for p53 or DNA-PK_CS_ from [*p53*^+/+^] HCT116 cells following Gem exposure for the time points indicated. + indicates 6 h pre-incubation with the ATM/ATR inhibitor CGK-733 (20 μM) or the DNA-PK inhibitor NU-7026 (10 μM). PCR was performed for the distal (-2.2 kb) *p21* promoter region. (B) ChIP assays for p53 or DNA-PK_CS_ were conducted as described in (A) and PCR was performed for the proximal (-1.3 kb) *p21* promoter region. (C) The quantification of the PCR bands shown in (A) and (B) and two repeated ChIP studies was carried out and normalized to each input lane. (D) ChIP assay for p53 or DNA-PK_CS_ from [*p53*^+/+^] HCT116 cells following Cr(VI) exposure for the time points indicated. + indicates 6 h pre-incubation with the ATM/ATR inhibitor CGK-733 (20 μM) or the DNA-PK inhibitor NU-7026 (10 μM). PCR was performed for the distal (-2.2 kb) *p21* promoter region. (E) ChIP assay for p53 or DNA-PK_CS_ was conducted as described in (D) and PCR was performed for the proximal (-1.3 kb) *p21* promoter region. (F) The quantification of PCR bands shown in (D) and (E) and two repeated ChIP studies was conducted and the values normalized to input samples as described in (C). The boxed areas highlight the effect of the ATM/ATR inhibitor on recruitment of early, but not late p53 to the *p21* promoter. Error bars for the graphs shown in (C) and (F) represent the standard deviation obtained from three independent experiments.

To test the possibility that the early p53 recruitment to the *p21* promoters could be mediated by ATM/ATR, ChIP analyses were carried out using the ATM/ATR and DNA-PK inhibitors. We found that the inhibition of ATM/ATR by CGK-733 delayed the early, but not the late recruitment of p53 to both the distal and proximal *p21* promoters under pro-death conditions (Fig. 5C and 5F, indicated on each graph in the boxed area). The temporal recruitment of p53 is now more in line with that of DNA-PK_CS_ which was unaffected by the inhibition of ATM/ATR. This result indicates that the early recruitment of p53 to the *p21* promoters is independent of DNA-PK_CS_ and mediated by ATM/ATR. Importantly, at later time points in the presence of sustained DNA damage there was the recruitment of DNA-PK_CS_ to the *p21* promoter-bound p53. The binding of both p53 and DNA-PK_CS_ to the *p21* promoters was effectively blocked by the DNA-PK inhibitor NU-7026, consistent with significantly attenuated p53 protein accumulation (Fig. 3B). A likely explanation is that the p53 that initially binds to the *p21* promoter at earlier time points becomes further modified at later times by DNA-PK_CS_ following its recruitment to the promoter.

RETRACTED

### DNA-PK_CS_ inhibition restores p21 expression and increases cell survival

We then questioned what the effect of DNA-PK inhibition would be on downstream p53-regulated genes under the various DNA damage conditions. Strikingly, repression of *p21* transcription following chromium or gemcitabine treatment was effectively reversed upon inhibition of DNA-PK, with the transcription of *p21* restored to levels comparable to those prior to damage (Fig. 6A) whereas inhibition of ATM/ATR had no effect suggesting that under these conditions DNA-PK_CS_ represses *p21* transcription. In contrast, under pro-arrest conditions (doxorubicin or IR), *p21* transcription was ablated when ATM/ATR was inhibited, whereas the inhibition of DNA-PK had no effect. This is consistent with the loss of p53 protein accumulation following the inhibition of ATM/ATR under pro-arrest conditions (Fig. 3B). In contrast to *p21*, chromium and gemcitabine exposure elicited an increase in both *PUMA* and *Bax* transcription (Fig. S7A) that was blocked by the DNA-PK inhibitor but not the ATM/ATR inhibitor. Enhanced expression of *PUMA* and *Bax* was also evident under pro-arrest conditions however this enhancement was ATM/ATR-dependent as it was blocked by CGK-733. As expected, in the absence of p53, there was little to no p53-regulated gene expression and that following treatment with each DNA damage modality there was limited transcription of these genes which was not significantly affected by ATM, ATR or DNA-PK_CS_ inhibition (Fig. S8B). It is noteworthy that these responses were conserved in a range of cancer cell lines (Fig. S7C and S7D).

**Figure 6:** Inhibition of DNA-PK_CS_ restores p21 expression under pro-apoptotic conditions (A) Trizol RNA extraction was carried out from [*p53*^+/+^] HCT116, A549 and Panc-1 cells 12 h post damage; cDNA was generated and the expression level for *p21* was measured. The mRNA expression levels were normalized to *GAPDH* mRNA, and are represented as fold increase or decrease over untreated cells. The DNA-PK inhibitor (NU-7026 [10 μM]) or the ATM/ATR inhibitor (CGK-733 [20 μM]) was pre-incubated for 6 h prior to DNA damage. (B) Immunoblot for p21, PUMA or Bax in [*p53*^+/+^] HCT116 cells 12 h post DNA damage. + indicates 6 h pre-incubation with the DNA-PK inhibitor NU-7026 (10 μM) or the ATM/ATR inhibitor CGK-733 (20 μM). For each gel β-actin indicates loading control. (C) Flow cytometric analysis of [*p53*^+/+^] HCT116 cells treated as described in (A). The percentage subG_1_ populations indicated in each FACS profile represent the average percentage from three independent experiments (10,000 total events counted per sample). (D) EC_50_ values were calculated using MTS assay for the [*p53*^+/+^] HCT116, A549 and Panc-1 cell lines 48 h post Cr(VI), Gem or Doxo treatment. The error bars for (D) represent the standard deviation obtained from three independent experiments.

RETRACTED

The protein expression levels under each DNA damage condition was also examined and was found to be consistent with our gene expression results (Fig. 6B). Following chromium or gemcitabine exposure there was the loss of the p21 protein. In contrast, there was significant accumulation of both PUMA and Bax. Inhibition of DNA-PK_CS_ restored p21 protein levels while reducing the levels of PUMA and Bax, consistent with our transcription studies. Furthermore, as predicted from our gene expression experiments, inhibition of ATM/ATR was unable to rescue the loss of the p21 protein and had no effect on the elevated PUMA and Bax protein levels. In contrast to chromium and gemcitabine treatment, both doxorubicin and IR exposure significantly increased the levels of all three proteins (p21, PUMA and Bax) in an ATM/ATR-dependent manner. Similar observations were made using the Panc-1 cell line (Fig. S8). Taken together, these observations are congruent with the notion that cell fate is dependent more on the regulation of expression of pro-survival genes (such as *p21*) than on the regulation of expression of pro-death genes (such as *PUMA* and *Bax*) and that DNA-PK and ATM/ATR play antagonistic roles in dictating these events.

To test this hypothesis we exposed cells to each damage agent in the presence of either the ATM/ATR inhibitor or the DNA-PK inhibitor. At 48 hours following Cr(VI) or gemcitabine exposure we note the significant accumulation of a sub-G_1_ population. In contrast and as predicted, doxorubicin or IR treatment induced cell cycle arrest (Fig. 6C). The inhibition of ATM/ATR did not significantly alter the sub-G_1_ population following Cr(VI) or gemcitabine treatment however as expected it did increase the sub-G_1_ population after doxorubicin or IR treatment [50, 51]. DNA-PK inhibition significantly reduced the sub-G_1_ population after Cr(VI) or gemcitabine exposure but had no discernable effect 48 hours post-doxorubicin or IR treatment. To complement our FACS approach we determined cell viability (EC_50_) for each chemical when ATM/ATR or DNA-PK was inhibited (Fig. 6D). In support of our data shown in Figure 6C, the inhibition of DNA-PK significantly increased cell viability after Cr(VI) or gemcitabine treatment but had no effect on cell viability following doxorubicin treatment. (We were unable to determine an EC_50_ value following IR treatment at 48 hours post damage). The inhibition of ATM/ATR did not significantly alter (although did lower) the EC_50_ for Cr(VI) or gemcitabine, however, it did cause a noticeable decrease (*P=*0.0259) in cell viability following doxorubicin treatment. In this regard it is interesting to note that a recent study showed that upon camptothecin treatment, ATM activation leads to cell cycle arrest, however when absent or inhibited, there is hyper DNA-PK_CS_ activation causing cell death [38]. We also addressed a previous report that demonstrated over expression of Myc can suppress *p21* transcription by forming a protein complex with Miz1 on the proximal *p21* promoter [52]. Our results indicate that the endogenous suppression of *p21* transcription following either gemcitabine or chromium exposure is DNA-PK_CS_ dependent and independent of Myc/Miz-1 (Fig. S9).

RETRACTED

## DISCUSSION

The present study reveals a mechanism whereby a key DNA damage sensor upstream of p53 is linked to a major effector protein downstream of p53, leading to cell death (Fig. 7). We demonstrate that under DNA damage conditions which induce p53-dependent cell death there is recruitment of DNA-PK_CS_ to the *p21* promoter. This promoter recruitment occurs by DNA-PK_CS_ binding to p53 on the p53 responsive elements within the *p21* promoter after DNA-PK_CS_ autophosphorylation. Upon DNA-PK_CS_ promoter binding, there is the rapid loss of *p21* transcription and the p21 protein. As a result of this ablated mRNA expression and subsequent protein loss, the cell is unable to induce cell cycle arrest and continues to cycle in the presence of sustained DNA damage. In striking contrast, under the same cellular conditions there is no DNA-PK_CS_ recruitment on pro-apoptotic promoters (*PUMA* or *Bax*) and consequently there is the elevated, continuous transcription of *PUMA* and *Bax*, producing a cellular environment that rapidly drives the cell towards apoptosis.

**Figure 7:** Model for DNA-PK_CS_-mediated repression of p21 transcription and induced cell death Under pro-arrest conditions (e.g. IR or Doxo), ATM/ATR is activated and modifies p53 promoting *p21* transcription and inducing cell cycle arrest. Concurrently, ATM/ATR phosphorylates DNA-PK_CS_, priming the latter for its DNA repair function. Under pro-death damage conditions (e.g. Cr(VI) or Gem), DNA-PK_CS_ undergoes autophosphorylation independently of ATM/ATR. DNA-PK_CS_ binds to p53 on the *p21* promoter, resulting in the abrogation of *p21* transcription. By preventing the accumulation of p21, DNA-PK_CS_ suppresses cell cycle arrest and p21-mediated survival, directing the cell towards cell death.

RETRACTED

A most important aspect of the present model is that it reconciles a number of key observations made through the years pertaining to the complex interplay between ATM, p53, p21, and importantly, DNA-PK, and amalgamates them into a single unifying mechanistic concept pertaining to the transcription regulation of *p21*. Under conditions that favor cell cycle arrest, the ATM/ATR signaling pathway is activated, triggering a p53 phosphorylation/acetylation cascade involving key p53 “arrest-specific” residues (e.g. phosphorylation at ser15 and ser315, and acetylation at lys382). Following *p21* promoter recruitment this “modified” p53 activates *p21* transcription, and cell cycle arrest ensues. Under pro-death conditions, the recruitment of DNA-PK_CS_ to the *p21* promoter apparently initiates a separate and different p53 phosphorylation/acetylation cascade (e.g. phosphorylation at ser15, ser37, ser46 and acetylation at lys120), which results in the abrogation of *p21* transcription. While precisely how the cell senses pro-arrest versus pro-death stress signals is unclear at present, a glimpse of the mechanisms involved in the transition from the pro-arrest to pro-death state could be gleaned from the time course experiment presented in Figure 5. During earlier times upon exposure to Cr(VI) or Gemcitabine, the recruitment of p53 to the *p21* promoter precedes that of DNA-PK_CS_, and that this recruitment is ATM/ATR-dependent. This “early bound” p53 likely functions as an activator of *p21* transcription, priming the cell for cell cycle arrest. Concomitantly, at these earlier times, DNA-PK_CS_ is phosphorylated, and this phosphorylation event is also ATM/ATR-dependent. It is tempting to speculate that the damaged cell is utilizing ATM/ATR to activate and couple p53's pro-arrest function with DNA-PK's DNA repair function. Indeed, recent evidence supports such a cross-talk between ATM/ATR and DNA-PK in situations where the repair of the damaged DNA is still a viable option [49, 53]. Under pro-death conditions, DNA-PK undergoes autophosphorylation, binds to and modifies p53 on the *p21* promoter, incapacitating p53's transcription activation function, and priming the cell to induce apoptosis by the ablation of *p21* expression. Although additional details will need to be worked out (e.g. the specific and sequential involvement of kinases and phosphatases, acetylases and deacetylases, and other p53 modifying enzymes etc.), the proposed model represents a general framework whereby ATM/ATR and DNA-PK are portrayed as key opposing players that dictate cell fate through the manipulation of a common switch, that of p53-mediated *p21* transcription.

RETRACTED

Our results lend credence to the intriguing notion that DNA-PK has dual roles, the first being its classically defined DNA repair role of mediating non-homologous end joining (NHEJ) and the second being its emerging role of driving apoptosis. It would seem logical to view these two roles as being mutually exclusive, which would in turn suggest the existence of a switch mechanism capable of exerting opposing biochemical and functional control of DNA-PK. While DNA-PK's DNA repair function necessitates its binding to broken DNA ends, the nature of putative DNA-PK binding to promoter elements is less clear. In this regard, it is noteworthy that signal-dependent activation of gene transcription has been shown to involve topoisomerase IIβ-dependent transient double strand DNA breaks with subsequent activation of poly(ADP-ribose) polymerase-1 (PARP-1) enzymatic function [54, 55], which could involve the recruitment of DNA-PK to the promoter site. While it remains to be seen how common DNA-PK-mediated transcription regulation through promoter binding occurs, the present study shows that the potential role of DNA-PK in apoptosis and cancer control cannot be understated and warrants further investigation.

## METHODS

### Cell lines and reagents

[*p53*^+/+^] HCT116 and [*p53*^−/−^] HCT116 human colon carcinoma cells were maintained in McCoy's 5A medium. A549 and Panc-1 human lung and pancreatic carcinoma cell lines were maintained in DMEM. All were supplemented with 10% FBS and antibiotics. Antibodies shown in supplemntal table 1 were used for our immunoblots and visualization of signal was achieved using an Odyssey^®^ Infrared Imaging System (Licor Bioscience, US). Doxorubicin (Sigma, US), gemcitabine hydrochloride (Eli Lilly #VL7502), chromium(VI) (potassium chromate (#03377 Sigma, US) were used at a concentration of 0.5 μM, 10 μM and 30 μM respectively. γ-Radiation (10 Gy) was delivered by a ^137^Cs gamma radiator (MDS Nordion) at 2.5 Gy min^−1^. Cells were pre-incubated with either the DNA-PK inhibitor NU-7026 (10 μM) or the ATM/ATR inhibitor CGK-733 (20 μM) (Tocris Bioscience, US) for 6 h prior to DNA damage.

### Cell viability (MTS) assay

Cells were seeded in 96-well plates at 1 x 10^4^ cells/well and 24 hr later treated with various DNA damaging agents Doxorubicin (Sigma, US), gemcitabine hydrochloride (Eli Lilly #VL7502), chromium(VI) (potassium chromate (#03377 Sigma, US) or γ-Radiation at the concentrations described. At the time points indicated post-treatment, cell survival was determined by CellTiter 96© Aqueous non-radioactive proliferation assay (MTS assay; Promega, CA, USA) following the manufactures guidelines.

RETRACTED

### Nuclear and cytoplasmic fractionation

Cells were washed once with ice cold PBS and then 1 ml of hypotonic lysis buffer (20 HEPES, 10 mM NaCl, 1.5 mM MgCl_2_, 0.2 mM EDTA, 20% glycerol, 0.1% triton X-100, 100 mM DTT, 1 mM AEBSF, 1 mM PIC) was added to each pellet. Nuclear fractions were harvested in hypertonic lysis buffer (20 mM HEPES, 500 mM NaCl, 1.5 mM MgCl_2_, 0.2 mM EDTA, 20% glycerol, 0.1% Triton X-100, 10 mM DTT, 1 mM AEBSF, 1 mM PIC).

### Co-immunoprecipitation

Co-immunoprecipitations (Co-IP) were performed as described in [34]). Cells were lysed in cold lysis buffer (50 mM Tris-Cl at pH 7.4, 150 mM NaCl, 1 mM EDTA, 1% NP-40, 0.25% sodium deoxycholate, protease inhibitor mixture). Cell extracts (500 μg) were incubated with the first antibodies (supplemental table S1) or control normal IgG on a rotator overnight at 4°C, followed by addition of protein G magnetic beads (Invitrogen, US) for 2 h at 4°C. Beads were then washed four times using the lysis buffer. The immune complexes were subjected to SDS-PAGE followed by immunoblotting with the secondary antibody.

### Western blot analysis

For the preparation of whole cell lysate, cells were harvested and lysed using RIPA buffer (50 mM Tris-HCl pH 7.4, 1% NP-40, 0.5% Na-deoxychlorate, 150 mM NaCl, 1 mM EDTA, 2 mM NaF, 2 mM NaVO_4_ and 1x protease inhibitor cocktail (PIC) (Sigma, US)). For SDS–PAGE, protein samples were boiled for 5–10 min in protein sample buffer (50 mM Tris pH 6.8, 1% SDS, 10% glycerol, 0.01% Bromophenol Blue, β mercaptoethanol [50 μL per 950 μL sample buffer]). Following electrophoresis, proteins were transferred onto nitrocellulose membrane (BioRad, US). The membrane was blocked for for 1 hour at room temperature or overnight at 4°C using 1X Odyssey® blocking buffer (Li-Cor, US). Primary antibodies were added to the membrane (supplemental table S1) overnight at 4°C or for 2 hours at room temperature. Secondary antibody was added (Licor, US) at typically 1:10,000 dilution for 1 hour at room temperature. Visualisation of signal was achieved using an Odyssey Infrared Imaging System (Li-Cor, US).

### Chromatin immunoprecipitation (ChIP)

Chromatin immunoprecipitation (ChIP) assays were performed essentially the same as described by Kaeser *et al* and Mattia *et al* [56, 57]. Briefly, cells were fixed with 1% formaldehyde, and then whole-cell lysates were prepared. Protein lysate was subjected to ChIP with the indicated antibodies (Supplemental table S1), followed by DNA purification. ChIP-enriched DNA was analyzed by PCR with the indicated primer sets (Supplemental Table S3). Visualization of bands was achieved using a Typhoon Phospho-imager (Amersham, UK) and quantified using the Image-Quant software (Amersham, UK).

RETRACTED

### Quantitative Real time PCR (qRT-PCR)

Total RNA was extracted by using Trizol (Invitrogen). Real Time PCR was performed on a Stratagene MX3000P PCR machine using the Stratagene Sybr® green master mix (Stratagene, Canada). The primer sequences for measuring p21, Bax, PUMA, MDM2 and GAPDH were purchased from Invitrogen and are shown in supplemental table S2. Data analysis was carried out using the 2^−∆∆CT^ method described by [58].

### Flow cytometric cell cycle analysis

Cells were grown to 60% confluence. BrdU was added to the medium 2 hours prior to DNA damage. Cells were mock treated/exposed to each DNA damage agent for 4 hours (in the presence of the DNA damage agent or following IR treatment). This corresponded to the 6 hour damage sample. Additional time points investigated were 0 hr (cells incubated in BrdU containing medium for 4 hours prior to sample collection), 2 hr, 12 hr, 24 hr and 48 hr. BrdU labeling was carried out utilizing an anti-BrdU-FITC antibody (Becton Dickinson) following the manufacturer's instructions. Samples were run on a Fluorescence Activated Cell Scanner (FACS) and the percentage with incorporated BrdU, the sub-G_1_ (non-viable apoptotic) population and the BrdU negative non-subG_1_ (viable) populations determined. 20,000 total events were scored per study BrdU was added to the medium 2 h prior to DNA damage. BrdU labeling utilizing an anti-BrdU-FITC antibody (#555627 BD Biosciences, US) was conducted and propidium iodide (2.5 mg mL^−1^) was added to the fixed, stained cells prior to analysis. 20,000 total events were scored per study from triplicate studies. Data was analyzed using FACS-express 3 (De Novo software, US).

### Statistical analysis

Statistical significance was assessed by one-way ANOVA or the two-tailed Students *t*-test. Statistical significance was defined as *P* < 0.05. Results are expressed as the mean ±SD.

## SUPPLEMENTAL INFORMATION

Supplemental information is linked to the online version of the paper on the Oncotarget website and includes supplemental figure legends, 9 supplemental figures (S1-S9) and 3 supplemental tables (T1-T3).

## Supplementary Figures and Tables




